This article has been retracted.

# A Modified LSTM Framework for Analyzing COVID-19 Effect on Emotion and Mental Health during Pandemic Using the EEG Signals

**DOI:** 10.1155/2022/8412430

**Published:** 2022-03-11

**Authors:** Aditi Sakalle, Pradeep Tomar, Harshit Bhardwaj, Md. Abdul Alim

**Affiliations:** ^1^CSE Department, Gautam Buddha University, Greater Noida, India; ^2^Department of Mathematics and Provost, Bangladesh University of Engineering and Technology, Dhaka, Bangladesh

## Abstract

COVID-19, a WHO-declared public health emergency of worldwide concern, is quickly spreading over the world, posing a physical and mental health hazard. The COVID-19 has resulted in one of the world's most significant worldwide lockdowns, affecting human mental health. In this research work, a modified Long Short-Term Memory (MLSTM)-based Deep Learning model framework is proposed for analyzing COVID-19 effect on emotion and mental health during the pandemic using electroencephalogram (EEG) signals. The participants of this study were volunteers that recovered from COVID-19. The EEG dataset of 40 people is collected to predict emotion and mental health. The results of the MLSTM model are also compared with the other literature classifiers. With an accuracy of 91.26%, the MLSTM beats existing classifiers when using the 70–30 partitioning technique.

## 1. Introduction

The COVID-19 epidemic has brought the world to a halt because of its rapid spread throughout the globe. Governments must impose lockdowns to stop the virus from spreading, which results in widespread social isolation, which can have serious mental illness repercussions [1]. The worldwide lockdown has affected people's livelihood and causes huge damage to their mental health. However, still, the resemblance of the effects of a pandemic on mental illness is not widely studied, and only little consequences have been identified. Given the significant links between pressure and the start of troubles among people's children due to emotion, it is critical to look at the impact that instructions to isolate themselves and stay at home are having on their mental illness [2]. During this time, it is critical to look into how individuals are concerned about becoming infected or suffering other COVID-19-related repercussions, and how this risk perception is changing [3, 4] and influencing their emotions, eventually leading to mental health issues [5].

It has been observed through research that the side effects of a pandemic on mental illness are regulated by different factors, such as age, networks in the society, occupation, responsibilities, financial condition, mental health problems, health issues, and personality behaviors [6, 7]. It should be a priority to investigate these connections since they are crucial in informing rules and healthcare choices, as well as guiding academics and physicians. However, there is a scarcity of information on how pandemics affect mental illness. Previous research on the association between COVID-19 and mental illness has focused on approximately restricted areas of mental health, failing to include the many psychosocioeconomic factors that are expected to alter impact, as well as the pandemic's negative-positive impact [8, 9].

To overcome this issue, we suggested a modified Long Short-Term Memory (MLSTM)-based Deep Learning model framework using electroencephalogram (EEG) signals for studying COVID-19's effect on emotion and mental health during the pandemic in this research paper. This research study was volunteered by participants who are detected with COVID-19 and recovered from it. In this study, we have tried to analyze the emotions of an individual by studying their brain waves using EEG signals which describe the mental health of individuals during pandemics. Emotion recognition-based behavior analysis benefits society and also it is an evolving research area [10, 11]. Emotion identification refers to a person's ability to recognize successful responses that occur in a variety of daily interactions. Awareness of emotional state can help society in many ways. For example, a person with a negative state of emotion can be given emotional help or medication if required and his or her emotional state can be improved, which further can improve their performance in society and at workplaces [12]. At the same time, the person with a positive emotional state can work for the welfare of society. The deployment of EEG signals to predict mental health has recently gained a lot of attention [13].

EEG signals have been more popular since they cannot be faked [14]. EEG signals reflect the electrical activity of neurons in the brain, and they have been frequently employed to study the working of the brain [15–18].

As it is difficult to counterfeit brain signals, in this paper, we are proposing a method that uses EEG for analyzing mental health during the pandemic. In this study, we have collected the dataset using an EEG device. The data captured with the help of EEG is nonmanipulative which is a major advantage in the research [19]. Explicit survey-based analysis of mental health and emotions during COVID-19 takes a lot of time, so this process needs to be automated so that a person can make the most of his/her potential and assistance can be provided to them to improve their mental health. The recording of brain signals directly cannot be falsified or disturbed. It helps in the detection of mental health to achieve a reasonable degree of precision because EEG is cheap, cost-effective, noninvasive, and speedy, making it a popular tool for testing brain changes to emotions. Using the NeuroSky MindWave Mobile 2 device, we have created the dataset by putting the electrode at the FP1 position because frequencies less than and larger than 0.5 Hz to 50 Hz, respectively, are not caught correctly [20, 21].

An MLSTM-based framework is developed for the analysis of COVID-19 effect on emotions and mental illness during the pandemic using EEG signals in this study. The 70–30 partitioning strategy is used to determine our model's performance. The results show that our model outperforms all other classifiers. This research includes the early detection of personality disorders, emotional distress, and other mental illnesses [22, 23]. During a pandemic, the psychological consequences are to improve people's quality of life and to maximize their performance [24, 25].

A short overview of this research work is as follows: (i) For analyzing COVID-19 effect on emotion and mental illness during the COVID-19 pandemic using EEG signals, a novel framework Deep learning-based modified MLSTM approach is proposed. (ii) A new EEG signal data collection (Dataset) is developed with an EEG portable single-channel computer-efficient platform for Indian emotional clusters in the Hindi language.

## 2. Proposed Work

In this section, the detail about the device used, dataset created, and the proposed algorithm is presented.

### 2.1. Device Stimuli Description

The NeuroSky MindWave Mobile 2 is a very cost-effective, portable, and easy to handle device. It captures the brain signals, and the components present in the device are flexible and long-lasting. The dataset required for this work is based on brain waves or EEG signals. These data are self-acquired using the NeuroSky MindWave Mobile 2 device, a single-channel EEG adjustable headband. The device outputs 12-bit raw brainwaves (1–100 Hz) with a sampling rate of 512 Hz and outputs EEG power spectra in different frequency and morphology bands.

The dataset is recorded using the eegId application, in which the FFT technique is implemented as a feature extraction method. A total of 10 features are extracted, referred as F1, F2….F10.

The EEG signals are generated as a person experiences different emotions or feelings when exposed to situations or scenarios through visual content. We recognize an individual's mental health by analyzing brain waves while watching emotional or situational materials and classifying the emotions into two classes, i.e., positive and negative. The elicitation materials included around 40 videos (Hindi-English languages). The defined process for data acquisition involves approximately 40 participants to watch precisely a set of 8 video clips that characterize real-life emotional experiences to analyze mental health. This recorded data of brain waves is processed, followed by applying deep learning-based and machine learning-based algorithms to study and analyze mental health during the pandemic and precisely predict the state of emotions.

### 2.2. Dataset

Forty (20 males and 20 females) nonclinical participants were considered for this research. The study was volunteered by participants detected with COVID-19 and recovered from it. The participants also signed an informed consent form. All nonclinical participants are from various cultures and education classes yet Hindi speaking. However, 5 data samples were dropped due to failure in equipment or excessive EEG signal artifacts in the final analysis. Therefore 35 samples were left as credible subjects (17 male and 18 female). The age group of participants is divided into three age groups 15–20 years, 21–26 years, and 27–35 years. The participants are divided according to their educational background as undergraduates, postgraduates, and working professionals. In our nonclinical population with healthy eyesight, two were left-handed and the remaining 33 were right-handed. Participants were instructed 24 hours before the experiment not to drink nicotine or caffeine. At the outstep, the context and process for the study were initially told to all participants in a manner consistent with the Helsinki Declaration definition. The experiment was performed twice with the same nonclinical population within one week.

Figure 1 explains the experimental protocol followed to create a brain signals dataset. A 10 sec hint was given to the participants to start the experiment. After watching the elicitation clips, the subject has to fill out the 3-point self-assessment form (1 = “agree”, 2 = “neutral”, and 3 = “disagree”) to rate the emotions. It consists of the binary class of emotions. Participants were urged to respond to their true feelings to all the questions.

### 2.3. Classification

In this study, the MLSTM model was employed to classify two classes of emotions (positive and negative) to analyze the effect of COVID-19 on mental health using EEG signals.

#### 2.3.1. MLSTM Architecture

Figure 2 shows the fundamental LSTM design. There are three gates in the modified LSTM network: a forget, an input, and an output. The MLSTM network uses these gates to decide what information to keep and remove from memory. Except for the hidden state, there is nothing else to recollect. Figure 2 reveals the network's secret. It shows the forget gate, which selects which information to keep and which cell states to discard. The choice is made with the help of the sigmoid layer.

(1) $$\begin{array}{c} f_{t}=\sigma \left(WT_{f}\cdot \left[h_{t-1},x_{t}\right]+b_{f}\right). \end{array}$$

The second gate with a sigmoid layer is the input gate, which determines values to be modified, and the layer tanh, which generates newly updated values.

Long EEG sequences are difficult to learn from a recurrent neural network because they are trained using time backpropagation (BPTT), which causes gradient disappearance. To tackle this problem, the recurrent neural network (RNN) cell is replaced with a port cell called the LSTM cell. Due to its reliance on subjective evaluations and EEG data categorization, MLSTM has no concept of gap length. Learning the long-term time-series dependencies and examining the temporal correlations of the EEG signals helps MLSTM achieve better outcomes when it comes to EEG signal categorization difficulties. MLSTM supremacy is also due to the model's explicit nature to prevent the long-term problem of reliance.

The MLSTM 1, MLSTM 2, and MLSTM 3 architectures are shown in Figure 3. Python 3.8 and TensorFlow 2.2.0 were used to build the MLSTM networks on the back-end. The simplest option is the MLSTM 1 design, which has 164 memory units in a single layer. The blocks of the memory store information, and these blocks are modified by three major processes, known as gates, which control the memory. Using the forget gate, it is possible to do what was left out of the cell state in the suggested way. The incoming EEG signal dataset is purged using the forget gate, which multiplies a filter. The MLSTM network must be optimized by making this change.

In the MLSTM_2 design, there is just one LSTM layer and a maximum of 268 memory units. A total of 732, 564, and 236 memory units are available in the MLSTM_3 architecture's three LSTM levels. There are 0.4 and 0.2 dropout layer probabilities. With dropout regularization, the MLSTM model has the advantage of better memorization without losing any of its core features. Overfitting is decreased, the model is trained quicker, and MLSTM model prediction performance is improved by employing the dropouts of 0.4 and 0.2. An activation function, known as “ tanh,” is used at the model's internal layer. Each of the three MLSTM networks has an output of 32, 56, and 64 units attributed by the “ tanh” activation function.

The “Softmax” activation function is utilized in the output layer to classify two types of emotions:

(2) $$\begin{array}{c} \text{Softmax}\left(x_{i}\right)=\frac{exp\left(x_{i}\right)}{\sum_{j}\exp\left(x_{j}\right)}. \end{array}$$

In our three MLSTM designs, overfitting was decreased by limiting unit coadaptation in the dropout layer. Categorical cross-entropy is the loss function in the dense layer for various network configurations. The Adaptive Moment Estimation optimizer (Adam) is used with a learning rate of 0.001. Using the MinMaxScaler function, the input attributes of the dataset are normalized. Each feature's contribution is consistent, thanks to this method's normalization. Network parameters vary during training, reducing internal covariate transition and shifting network activation distribution. Internal covariance change is reduced as a result of network normalization. Ping weights were also restricted to prevent them from expanding throughout the whole site due to the optimization procedure. The mechanism becomes more regular due to normalization, which was not the desired outcome. 1000 iterations with 40 batch sizes were used to evaluate the proposed model's output. The gathered EEG dataset was used to evaluate each MLSTM prototype. Based on our trials with nearby architecture, we selected these buildings and qualities (in terms of layers and nodes). Because they outperform their nearby design in terms of accuracy throughout 500 epochs, these three structures were considered in our analysis. According to the correctness of the MLSTM_3 architecture, Table 1 presents the assessment results on several epochs. The parameters for evaluating performance will be explained in the next section.

## 3. Performance Measure

The MLSTM architecture is analyzed by calculating the accuracy, recall, precision, and Mann–Whitney test performance measures.

### 3.1. Accuracy

It is the ratio of corrected samples to the total samples:

(3) $$\begin{array}{c} \text{accuracy}=\frac{TP+TN}{TP+TN+FP+N}\times 100. \end{array}$$

### 3.2. Recall and Precision

Recall and precision can be given as

(4) $$\begin{array}{c} \text{recall}=\frac{TP}{TP+FN}, \end{array}$$

(5) $$\begin{array}{c} \text{precision}=\frac{TP}{TP+FP}. \end{array}$$

### 3.3. Specificity

It is the ratio of true negative to the true negative plus false positive:

(6) $$\begin{array}{c} \text{specificity}=\frac{TN}{TN+FP} \end{array}$$

### 3.4. Mann–Whitney Test

Mann and Whitney [26] test can provide the significant difference of the samples. It calculates the *p* values of the model and describes its effectiveness.

## 4. Results

The result of the proposed architecture is presented in this section. The details of the device used for implementing all the models MLSTM_1, MLSTM_2, MLSTM_3, MLP, KNN, SVM, LibSVM, and CNN are Intel 5, 16 GB RAM, 1 TB hard disk, and the language used for implementing all the models is Python. The parameter values for implementing the MLP, KNN, SVM, LibSVM, and CNN models are taken from [27–31], respectively. The parameter values used for implementing the MLSTM architectures are dropouts of 0.2 and 0.4, Adam optimizer, 0.001 learning rate, 500 epochs (best accuracy achieved but trained till 1000 epochs).

The 70–30 partition is used to evaluate the performance. In this, 70% of the sample is kept in training data and 30% is used for testing the architecture. All the performance measures are calculated using this partition scheme, demonstrating the results.

### 4.1. Evaluation of the MLSTM Architecture

The three deep learning MLSTM architecture has been implemented in the research for two classes of emotion classification to analyze the mental state during the pandemic with EEG signals. To show the dominance of the LSTM [11] architecture, it has been compared with the ML models. It is proved from the literature that due to the presence of computational and classification unit, LSTM architecture showed superiority over ML models that is also confirmed from our results. The ability to handle the sequential and time-series data makes them one of the best choices for emotion recognition.

Table 2 describes the accuracy of two classes of emotion classification to analyze the mental state during the pandemic with EEG signals among 3 MLSTM architectures. The MLSTM_1 gets the 63.76%, 60.24%, and 57.87% maximum, average and minimum accuracy, respectively, for the 70–30 partition scheme.

The MLSTM_2 acquired the 77.43%, 74.34%, and 70.19% maximum, average, and minimum accuracy, respectively. This is much higher than the MLSTM_1 architecture.

The MLSTM_3 architecture has the best accuracy among all the architecture. The maximum, average, and minimum accuracy achieved is 91.26%, 88.92%, and 85.18%, respectively. This confirms that MLSTM_3 is the best among the three architectures.

Figure 4 represents the accuracy as compared to the training loss. The loss calculation is done by calculating the difference between actual and predicted values. The loss function used here is categorical cross-entropy, as it is one of the most used loss functions.  Figure 5 represents the accuracy as compared to the testing loss. It is clear from the graph that the model has an average accuracy of almost 90% with minimal loss, which shows the superiority of our model for emotion recognition.

## 5. Discussion

Table 3 describes the performance of the model in terms of accuracy. The results show that MLSTM_3 architecture outperforms the other two architectures.

A comparison of the proposed architecture with the other machine learning models is made. All the models used in this study are implemented using the same set of features. The environment for developing the model is also the same that gives a fair comparison of the work.

The accuracy of MLP is 75.34%, the accuracy of KNN is 72.42%, the accuracy of SVM is 78.23%, the accuracy of LibSVM is 81.72% the accuracy of CNN is 79.72%, and the accuracy of MLSTM_3 is 91.26%. The accuracy of the proposed architecture is almost 10% higher than the second-best model that showcases the effectiveness of MLSTM_3 architecture.

The other performance measures are described in Table 4. It is clear from the result that MLSTM_3 architecture has very low false-positive and false-negative rates. That is also very significant in terms of measuring the model performance.

Table 5 presents the Mann–Whitney test [26]. The *p* value describes the significance of the model with other models. If the *p* value is larger than highly significant, their low *p* value describes the insignificance of the architecture. Here, all the values are highly significant, which is very important in measuring the model.

## 6. Conclusion

In this paper, an MLSTM architecture for two classes of emotion classification to analyze the mental state during the pandemic is proposed. We have collected a dataset of 40 people for doing the emotion classification. Also, the MLSTM architecture was developed to classify positive and negative emotions; the results ensure that it outperforms all other methods for emotion classification. The limitation of this work is that we have used a 1-channel EEG device for data collection. It will be interesting to analyze the result of other EEG devices like 4-channel, 14-channel, and 16-channel. In the future, we want to create a more extensive dataset and analyze our result on more participants that may help our classifier to improve.

## Figures and Tables

**Figure 1:** EEG experiment protocol.

**Figure 2:** LSTM cell network architecture.

**Figure 3:** Three MLSTM cell network architecture.

**Figure 4:** MLSTM_3 model accuracy and training loss plot.

**Figure 5:** MLSTM_3 model accuracy and testing loss plot.

**Table 1:** MLSTM_3 model accuracy on various epochs.

Epochs	Accuracy
300	87.44
400	89.38
500	91.26
600	90.82
700	89.95
800	89.17
900	88.84
1000	88.04

**Table 2:** Classification accuracy comparison of MLSTM classifier's for mental health analysis during pandemic by classifying two classes of emotions.

Method	Validation technique	Accuracy		
		Max	Avg	Min
MLSTM_1	70–30	63.76	60.24	57.87
MLSTM_2	70–30	77.43	74.34	70.19
MLSTM_3	70–30	**91.26**	**88.92**	**85.18**

Bold shows the maximum, average, and minimum accuracy values in percentage obtained when MLSTM_3, the proposed classifier, is applied for data classification.

**Table 3:** MLSTM_3 vs other ML models.

Method	Partition	Accuracy		
		Max	Avg	Min
MLP	70–30	75.34	72.66	69.53
KNN	70–30	72.42	70.12	68.86
SVM	70–30	78.23	76.53	74.58
LibSVM	70–30	81.72	79.42	77.46
CNN	70–30	79.72	75.28	72.99
MLSTM_3	70–30	**91.26**	**88.92**	**85.18**

Bold shows the maximum, average, and minimum accuracy values in percentage obtained when MLSTM_3, the proposed classifier, is applied for data classification. The table compares accuracy values when ML models are used and when the proposed classifier is applied.

**Table 4:** Sensitivity, precision, and specificity values.

Partition classifier MLSTM_3			
	Sensitivity (%)	Precision (%)	Specificity (%)
	Mean ± std	Mean ± std	Mean ± std
70–30	**90.46**±**2.14**	**89.63**±**2.28**	88.74 ± 2.34

Bold shows the sensitivity, precision, and specificity values in percentage obtained from the confusion matrix when 70 percent data are used for training, 30 percent data are used for testing and MLSTM_3, and the proposed classifier is applied for data classification.

**Table 5:** *p* value for MLSTM_3.

		MLP		KNN		SVM		LibSVM	
		*p* value	Significance	*p* value	Significance	*p* value	Significance	*p* value	Significance
MLSTM_3	70-30 partition	2.551 1 × 10 ^−13^	Highly significant (HS)	1.350 × 10^−13^	HS	1.870 3 × 10^−13^	HS	1.986 3 × 10^−13^	HS

## Data Availability

The data are available on request from the corresponding author.
